RETRACTED

# Vehicle Safety-Assisted Driving Technology Based on Computer Artificial Intelligence Environment

**DOI:** 10.1155/2022/4390394

**Published:** 2022-06-18

**Authors:** Haibo Yan

**Affiliations:** Macau Institute of Systems Engineering, Macau University of Science and Technology, Macau 999078, China

## Abstract

In this paper, we propose an assisted driving system implemented with a Jetson nano-high-performance embedded platform by using machine vision and deep learning technologies. The vehicle dynamics model is established under multiconditional assumptions, the path planner and path tracking controller are designed based on the model predictive control algorithm, and the local desired path is reasonably planned in combination with the behavioral decision system. The behavioral decision algorithm based on finite state machine reasonably transforms the driving state according to the environmental changes, realizes the following of the target vehicle speed, and can take effective emergency braking in time when there is a collision danger. The system can complete the motion planning by the model predictive control algorithm and control the autonomous vehicle to smoothly track the replanned local desired path to complete the lane change overtaking action, which can meet the demand of ADAS. The path planner is designed based on the MPC algorithm, solving the objective function with obstacle avoidance function, planning the optimal path that can avoid a collision, and using 5th order polynomial to fit the output local desired path points. In 5∼8 s time, the target vehicle decelerates to 48 km/h; the autonomous vehicle immediately makes a deceleration action and gradually reduces the speed difference between the two vehicles until it reaches the target speed, at which time the distance between the two vehicles is close to the safe distance, obtained by the simulation test results. The system can still accurately track the target when the vehicle is driving on a curve and timely control the desired speed change of the vehicle, and the target vehicle always maintains a safe distance. The system can be used within 50 meters.

## 1. Introduction

The advent of the automobile has had many effects on people's lives. It has made people's travel much more efficient. In the past, places that seemed to be out of reach have become less distant with the development of road traffic and automobiles. With the passage of time and rapid economic development, cars have become more popular. In the old society, only a scattered number of cars could be seen on the streets, but in today's modernized world cars have penetrated almost every household as an important means of transportation. But, with the increasing number of cars, and with it, the road danger index has increased exponentially. Therefore, the safety of automobiles is an important research point in front of people. According to the World Health Organization, traffic accidents have become the second leading cause of death among young people and the third leading cause of death among young and middle-aged people in the world [1]. The assisted driving system is such an active safety system, which can monitor road information and driving conditions in real time, can automatically identify traffic warning signs for prompting or warning, can determine whether the distance to the traffic ahead is within the safe range, whether there is a possibility of collision, can determine whether the local cars or pedestrians are within the safe range, and can determine whether the driver is driving in fatigue. In case of danger, he will take over the driving right and take the initiative to brake to avoid the accident.

RETRACTED

From ITS to intelligent transportation, both theory and application represent the progress of society, and vigorously developing intelligent transportation is an important part of building a sustainable country in China. People's travel experience and the traditional old way of travel, which is conducive to the sustainable development of society, are an important way to improve the national standard of living [2]. Future transportation will develop towards the trend of increased automation and more intelligence. At present, the technologies strongly advocated by the traffic management department are vehicle-vehicle communication and vehicle-road communication based on vehicle-road cooperation technology, vehicle sensing system based on video recognition and frequency projection technology, and automatic driving system [3]. In this paper, with the background of building a scientific intelligent transportation system, we select road intersections with complex traffic environments as the main research object and research traffic flow control model and algorithm of road intersections under the background of intelligent transportation.

For the traffic sign recognition module, image processing techniques are used to perform image enhancement on the extracted images and segmentation of the targeted traffic sign region in the enhanced images. Convolutional neural networks are used as classifiers to train the dataset and image enhancement techniques are used to expand the relevant dataset. Finally, training and analysis are performed on the host platform. The pedestrian detection module is trained for the pedestrian dataset using a convolutional neural network, which includes the expansion of the dataset with annotation, and finally the simulation verification operation is performed with the camera through the embedded platform, and the training results are analyzed. Finally, an unmanned vehicle assisted driving system including traffic sign recognition and pedestrian detection is designed, its basic process is designed, and both traffic sign classification and pedestrian detection parts are implemented and analyzed. Ground segmentation based on LIDAR point cloud features based on ray slope thresholding method is performed to obtain the road passable area, which is compared and analyzed with the planar model segmentation method based on random sampling consistency. For the vehicles driving on the highway, the point cloud clustering process is based on Euclidean distance, the state estimation of the clustered targets is performed by interactive multimodal probabilistic data matching and traceless Kalman filtering algorithm to realize the tracking of target vehicles, and the effectiveness of the algorithm is verified by real point cloud data. Design vehicle safety assistant driving technology using artificial intelligence driving technology algorithm.

RETRACTED

## 2. Current Status of Research

Abraham et al. designed a system called AutoGuide, and the underlying prediction applied a historical averaging model [4]. The advantage of the historical averaging model is its simple calculation principle and low complexity, but it does not reflect enough the dynamic characteristics and nonlinear features of traffic flow, so it cannot be applied to the field that requires more accurate prediction results [5]. Currently, this type of method is mostly used in the replacement of lost data and has achieved good results. Weiss et al. first applied Kalman filtering to the prediction of actual traffic flow and compared the results with the historical averaging method, which showed that the accuracy of the filtering algorithm was higher than that of the historical averaging method [6]. The results showed that the accuracy of the filtering algorithm was higher than that of the historical average method. At the end of the same year, Ledezma-Zavala et al. designed a traffic flow prediction model based on Kalman filtering with the data collected by sensors to better predict the traffic flow of highways [7]. The research of these intelligent vehicles is mainly to add various detection devices to existing vehicles, using these detection devices to collect the environmental conditions, and through the computer to calculate and integrate and then issue control commands to guide the vehicle driving [8]. The whole system is equivalent to a mobile processing system to perform automatic control tasks [9]. The system is still in the testing and exploration phase and human intervention is still required [10]. This is due to the complexity of the actual operating environment and the occurrence of unexpected events that can cause the machine to produce a slight deviation, because the machine is ultimately a machine, even if the machine can respond to some fixed elements, but up to some perceptual elements it will be incompetent, and artificial intelligence to detect fixed elements still has detection errors but also needs a longer time to explore it [11]. The car has landed, but the technology has not yet been completely conquered and can be popularized in daily life which is still too early [12]. In response to these safety issues, our focus is still to concentrate on the auxiliary driving system, which includes automatic parking, collision warning, cruise control, range radar, GPS navigation, and lane departure control.

RETRACTED

According to the control mode, the timing model of road intersections can be divided into a single-point control model and arterial cooperative control model [13]. Using the advantages of fuzzy control and Q-learning algorithm, Korssen et al. proposed a hierarchical control model to realize the cooperative control of road intersections [14]. The calculation of the green signal ratio and period of each intersection in the next cycle is done at the control layer, while the adjustment of the arterial phase difference is realized at the coordination layer using the Q-learning control method, which significantly improves the average driving speed of vehicles and greatly reduces the delay time compared with the commonly used timing scheme and the traditional genetic algorithm-based timing scheme [15]. Uchida et al. designed a discrete mathematics-based trunk line coordination control model, divided the delay calculation of trunk lines into two parts, external import lanes and internal import lanes, proposed a multiobjective optimal signal timing model for trunk line cooperative control, and used a genetic algorithm to solve it [16]. Biondi et al. designed a parameter dynamic adjustment strategy to better optimize the coordinated control of two-way traffic signals on trunk lines, and this model is based on the standard difference (P-ADE) algorithm [17]. The balance between global search and local search is ensured, and the results show that the advantages of this method in terms of algorithm speed, accuracy, and robustness are obvious. In the same year, Song et al. first designed a multiobjective optimization model for signal coordination control based on multiple intersections to consider multiple objectives and then designed a new solution algorithm by modifying the nondominated ranking genetic algorithm to realize the solution of the multiobjective optimization algorithm [18].

RETRACTED

The current research on basic issues such as the method of phase switching decision and the phase structure is still lacking, and the research on the system of single-point and arterial signal coordinated control still cannot meet the requirements of social development. In addition, most of many arterial coordination control algorithms currently proposed cannot meet the requirements of the actual traffic scenarios for algorithm in real time. Vehicle collision avoidance technology is based on the use of satellite, radar, video detection, and other technologies to achieve real-time sensing of driving vehicle information, using computers to analyze and process the sensed information, and apply the results to the driving vehicle's auxiliary driving or automatic driving, using steering angle or brake braking and other control methods to achieve collision avoidance between the target vehicle and the conflicting vehicles. The existing collision avoidance algorithms and models mainly include probabilistic and mathematical statistics-based motion trajectory estimation models, models based on vehicle-road cooperation technology or vehicle-vehicle communication technology, models based on intelligent learning, models based on optimal control technology, and kinetic collision avoidance models.

## 3. Analysis of Automobile Safety-Assisted Driving Technology in the Artificial Intelligence Environment

### 3.1. Artificial Intelligence Driving Technology Algorithm

Vehicle recognition is a prerequisite, and the sensors that can be used are monocular vision, stereo vision, millimetre-wave radar, and multisensor fusion. At present, vehicle recognition based on monocular vision grayscale images is the most widely researched and involves more algorithms, and the famous ADAS company Mobileye is using monocular vision solutions to solve the problem. Vehicle detection generally relies on vehicle feature information, such as vehicle shape and. the ratio of vehicle height to vehicle width, as constraints for detecting vehicle edges, and edge enhancement processing is performed on the image to obtain some horizontal and vertical edges containing vehicle information, to detect the vehicle. The algorithm using a monocular camera is simple and the computation is done in real time, but the monocular vision scheme is susceptible to external environmental factors such as lighting and shadows, which make it less reliable. Stereovision is another path that has emerged in recent years, directly simulating the way human vision processes scenery by observing the same scene from multiple viewpoints to obtain perceptual images under different perspectives. Existing stereovision technology is not quite mature and the research is much less enthusiastic than monocular vision. In addition, in order to break through the limitations of a single sensor, the use of multisensor information fusion technology is also the mainstream of current research. The common vision and laser sensor fusion and vision and millimeter wave radar sensor fusion have the disadvantages of high cost and more complex calculation, resulting in poor real-time performance.

RETRACTED

Classification problems focus on what objects the icon primarily describes and how the object is classified. The localization problem, on the other hand, finds this object on top of the classification. And when there are more targets in the picture, it is not possible to perform a single classification, but a multiobjective task. Finding the position of each target among multiple targets and writing an accurate classification is the target detection problem. And the problem of wishing to label the targets in the picture by pixels is the semantic segmentation problem. The R-CNN as a landmark network for target detection: first, the model input is a picture, then about 2000 regions to be detected are proposed on the picture, then these 2000 regions to be detected are extracted features one by one (in series) by the convolutional neural network, and then these extracted features are classified by a support vector machine (SVM) to obtain the class of the object and resize the target enclosing box by a wraparound box regression computation module.

Bilateral filtering is a common filtering method, which is a nonlinear filter. It is a compromise process that combines two factors, spatial proximity and pixel value similarity, while considering the space domain location information and pixel similarity, so that it can achieve the effect of removing image noise again without destroying the image edge information [19]. However, other filtering methods, such as mean filtering and Gaussian filtering, are difficult to do them. The specific principle is that bilateral filtering has one more Gaussian Sigma-d variance based on spatial distribution than Gaussian filtering, so that edge pixels and nonedge pixels do not affect each other. However, it also has the disadvantage that this filtering of high-frequency information is not significant due to the excessive high-frequency information of its filter and it can only filter low-frequency information better [20]. In the bilateral filter, the value of the output pixel depends on the combination of the weighted values of the neighbouring pixel values,

(1) $$\begin{array}{c} g\left(i,j\right)=\frac{\sum_{k,l}f\left(k,l\right)w\left(i,j,k,l\right)}{\sum_{k,l}f\left(k,l\right)}, \end{array}$$

and the weighting factor *w*(*i*, *j*, *k*, *l*) depends on the product of the null domain kernel and the value domain kernel. (*i*, *j*) and (*k*, *l*) refer to the coordinates of two-pixel points, respectively. The airspace kernel is expressed as follows:

(2) $$\begin{array}{c} d\left(i,j,k,l\right)=\exp\left(\frac{{\left(i+k\right)}^{2}-{\left(j+l\right)}^{2}}{2\sigma_{d}^{2}}\right). \end{array}$$

The value domain kernel is expressed as

(3) $$\begin{array}{c} r\left(i,j,k,l\right)=\exp\left(\frac{{\left(i+k\right)}^{2}+{\left(j+l\right)}^{2}}{2\sigma_{r}^{2}}\right). \end{array}$$

Multiplication of the two results in a data-dependent bilateral filtering weight function.

(4) $$\begin{array}{c} w\left(i,j,k,l\right)=\exp\left(\frac{{\left(i+k\right)}^{2}+{\left(j+l\right)}^{2}}{2\sigma_{d}^{2}}-\frac{{\left(i+k\right)}^{2}+{\left(j+l\right)}^{2}}{2\sigma_{r}^{2}}\right). \end{array}$$

The *D* function selects the weights based on the pixel distance. This is the same as the box filter and the Gaussian filter. It has a greater proportion of pixel value similarity than the distance factor between pixels. The function, on the other hand, maintains the edge characteristics; i.e., the differences can be large even if the pixels are close to each other [21]. Image smoothing is the process of removing noise. Most parts of the image are mainly concentrated in the low-frequency part, while the noise is mainly concentrated in the high-frequency part. But the edge information of the image is also in the high-frequency part. So, after the smoothing process, some edge information will be lost. So, we need to use the sharpening technique to enhance the edge information. Smoothing is sharpening the image after using differential or integral operations. And the differential operation is the calculation of the rate of change of the signal, and it can effectively increase the high-frequency component. And, before sharpening the image, we must make sure that the image has high-frequency information; otherwise, there will be a lot of noise after image processing.

RETRACTED

The essence of the brightness contrast of an image is to adjust the pixels of the image iteratively, by adjusting the gray level of the pixels to adjust the overall brightness of the image, and the contrast is mainly the size of the color difference between the black and white colors in the image.

(5) $$\begin{array}{c} g\left(x\right)=af\left(x\right)-\beta . \end{array}$$

The parameter *α* is called gain and parameter *β* becomes bias. We often use these two parameters to control the brightness and contrast. *f*(*x*) is the input of the function; i.e., the pixel of the input image *g*(*x*) is the output of the function, i.e., the pixel value of the insights after processing, and the above formula can be refined to the following function.

(6) $$\begin{array}{c} g\left(i,j\right)=\alpha f\left(i,j\right)-\beta , \end{array}$$

where *i* indicates that *j* pixels are in row *i* and column *j*. *α* adjusts the contrast of the image and *β* adjusts the brightness of the image.

Our real world is colourless, and the reason why we can see colors is because of the presence of light, which shines on objects and then reflects our eyes to form the images that we see. For example, water is colorless, but the water film has color because it can reflect, while water can only refract. Virtually, all colors are composed of the three primary colors, red, green, and blue. The basic principle of the retinal theory is that the presentation of an object's color depends on various linear combinations of its reflected long (red), medium (green), and short (blue) waves, rather than on the intensity of the reflected light. Objects are affected by the consistency of light; i.e., Retina is based on the consistency of color perception and, in contrast to traditional nonlinear methods, Retinex can compensate for dynamic range compression, perform edge enhancement, and adjust color constants to adaptively improve different types of images. In the last 40 years, researchers have developed retinal algorithms based on the human visual system, from single-scale retinal algorithms to multiscale weighted average MSR algorithms and finally to color recovery multiscale MSRCR algorithms, and then to retinal algorithms. Retime algorithms are useful for images with brighter images by suppressing high luminance and enhancing color components on the image. The general Retinex algorithm assumes that the initial illuminated image is slowly changing when estimating the illuminated image; i.e., the illuminated image is smooth.

There are many algorithms for detecting triangles with the Hough transform, but this paper uses one for detecting triangles by first detecting the target boundary, then creating a regression function by which a specific model is created, and if the model satisfies the conditions of the triangular shape, then detected Figure 1 is a triangle. The method first transforms the image using the Hough transform and then locates the triangle formed by detecting the straight-line segments that satisfy the triangle condition. After analysis, the Hough transform can not only detect circles but also be applied to detect straight lines. For triangular traffic signs, which are composed of three regular line segments, the Hough transform can also play a role in detecting the effect, as shown in Figure 2.

RETRACTED

This is a mandatory step before training all neural networks. The purpose of training our neural networks is actually to bring the weights on the neural network to the values that we expect, which are often unknown. In an untrained initial network, the weights will certainly not match our expectations. So, how do we set these parameters? Generally, we fix a rough range to randomize these network parameters so that they follow a certain probability distribution, and this method is called weight initialization.

The concept of learning rate is built under the propagation algorithm of gradient descent. The complexity of our neural network can be defined as a loss function *G*(*x*), which symbolizes the error that exists between the predicted value and the true value, and our goal is to make it 0. Gradient descent is a method that can reduce the value of the loss function, and it is a way that utilizes the downhill style, where each input batch of images the gradient descent is a method that reduces the value of the loss function by using a downhill approach in which the gradient and step size are calculated once for each input batch of images, and the value of the loss function is reduced by this gradient and step size. And the learning rate then affects the step size of the descent. Generally speaking, the larger the learning rate, the faster the loss function decreasing, and the faster the network fitted, but the accuracy is not high. In contrast, the training strategy with a small learning rate step is more accurate, although the iterations are slower.

(7) $$\begin{array}{c} L_{\text{IOC}}\left(t^{k},v\right)=\sum_{i\in x,y,w,h}{\text{smooth}}_{L_{1}}\left(t_{i}^{k}+v\right),\\ L\left(p,k,t^{k},v\right)=L_{cLs}\left(p,k\right)-\lambda \left[k\leq 1\right]L_{\text{IOC}}\left(t^{k},v\right). \end{array}$$

The constraint *k*=0 indicates the background, which is not involved in the calculation of the cost function of the border regression. The input of the region of interest proposal network is the feature map output from the convolution part of the neural network, corresponding to two outputs, which are the location information of the region of interest, i.e., a quadratic array and the category of the candidate region, where only a binary classification is done to determine whether the region is a background or a target. To get these two outputs, the RPN network needs to get the position information of the region of interest in the input image and the feature maps corresponding to each region of interest.

RETRACTED

### 3.2. System Experimental Design

The software of the auxiliary driving unit adopts a modular design, including the initialization module and CAN communication module. The initialization module is mainly responsible for the power-on initialization of the auxiliary driving unit, initializing and setting the XC2287M, the main controller chip of the auxiliary driving unit, configuring the control registers of the XC2287M chip, enabling the CAN nodes, and finally calling the CAN communication module, which configures the CAN register of the XC2287M, sets the CAN nodes and message objects, and communicates with the car CAN bus through the CAN communication module configures the CAN register of XC2287M, sets the CAN nodes and message objects, and communicates with the car master through the car CAN bus to realize the design function of the assisted driving unit. The software design scheme of the auxiliary driving unit is shown in Figure 3.

The XC2287M provides a 16-bit watchdog timer to check the software and hardware for faults, and the watchdog will reset the XC2287M system if the system does not operate the watchdog for a certain period. After the initialization module is completed, the CAN communication module is called, and its functions include CAN node initialization, message object initialization, CAN transmitter module, CAN receiver module, distance information processing, and error processing. After the CAN node is ready, the auxiliary driving unit joins the CAN bus of the vehicle and participates in CAN communication. The communication program mainly hands over the frames prepared by distance information processing or error processing to the sending function module for sending or uses the receiving function to receive information from the CAN bus.

The problem that segmentation networks are difficult to be practical is even bigger. Pixel-level segmentation, because it is specific to each pixel, also makes the classification of pixels with a higher error rate. The decision module needs to understand the location of its situation and the precise positioning of the environment in the surrounding scene. Segmentation can lead to many additional decision errors, most misclassified noise in the drivable area [22]. This misclassification cannot be left unaddressed for safety reasons and is handled in as conservative a manner as possible for safety reasons; otherwise, the Uber self-driving vehicle crash would result in irreversible loss of life and social confidence in the application of self-driving technology.

The characteristics of these different models need to be selected for a specific problem. The partial structure of the different models is drawn and integrated to achieve an effective model for a specific problem. In real vehicle test environment scenarios, decision-based evaluation metrics are what should be proposed and applied. And different neural network learning criteria should also be selected in different domains. This is not yet practical on a large scale in the current applied technology. This is because the current imprecise perception in autonomous driving is also sufficient to accomplish the work in low-speed scenarios. With safety in mind, all imprecision can be temporarily ignored altogether. With the help of lidar, the program design also gives more accurate data to the local environment. Even at a greater cost, it is impossible to completely replace the camera. It can be said that this is still vision technology which is not stable and reliable enough. It is also the reason why deep learning technology cannot be fully trusted although it is considered the main core technology of the future and a certain scale of experimentation, as shown in Figure 4.

RETRACTED

The dataset contains real image data collected from urban, rural, and highway scenes, with up to 15 vehicles and 30 pedestrians per image, as well as various levels of occlusion and truncation. The entire dataset consists of 389 pairs of stereoimages and optical flow maps, 39.2 km visual ranging sequences, and over 200 k images of 3D annotated objects, sampled and synchronized at 10 Hz. The dataset data acquisition platform includes 2 grayscale cameras, 2 color cameras, a Velodyne 3D LIDAR, 4 optical lenses, and a GPS navigation system.

It can be seen that the detection effect does not decrease significantly in the multitask network. The multitask model whose segmentation effect is compared with the semantic segmentation network is shown in Figure 4. It can be seen that there is a more significant decrease in the accuracy rate. With the Kitty dataset, the target detection effect can reach about 80%. The IoU parameter hovers around 50%. Since the multitasking network is mainly based on the target detection network, it can be seen from the data that the multitasking network has a better detection effect [23, 24]. Because the method ignores the edge details of the drivable area, the segmentation effect is lower as expected.

## 4. Analysis of Results

### 4.1. Artificial Intelligence Algorithm Results

Data analysis and processing cannot be done without an understanding of the problem; otherwise, the data is just a cold structured data mass and cannot bring effective knowledge. The analysis of the data here is mainly focused on the analysis of the data of the width of the vehicle. This is because, in real scenarios, vehicles are generally moving in the direction of the road, so the focus is generally on the forward target, and the most useful place for the camera is precisely the understanding of the forward target at medium and long distances. Then, the practical problem is that in more scenarios, the main target is the rear view of the forward facing vehicle. And the distance detection approach proposed in the next section is also based on the width of the forward-facing vehicle for processing, which will be described in the next section. However, because the flow in the subsequent work is needed, the focus in this chapter is also on the mapping relationship between the width information of the vehicle model and the vehicle model. The second focus will also be on the relationship between vehicle length and model. However, this is the data that is quite discrete in the initial processing. The model length and width correspond to Figure 5, and it can be seen that there is no fixed distinguishable distribution of all the statistics of the model width. The distribution of the length and width of different types of models is also discrete, and although the aspect ratio of vehicles seems to have a relatively clear upper limit, its distribution is still mixed and messy.

RETRACTED

The results of the experiments in this chapter are shown in Figure 6. As can be seen from the table, the effect of model compression is very significant, as this method is 10 times smaller than the compressed AlexNet model, while the average accuracy (mAP) is 0.4% higher than that of the compressed AlexNet model, which is only 350 times smaller than that of the uncompressed AlexNet network. Because of the more complex composite bypass structure, this method is 0.2 MB larger than the compressed Squeeze Net but has better detection results.

The average IOU metric of training symbolizes the average deviation of the predicted bounding box from the true bounding box, ideally, 100%; i.e., the output bounding box exactly coincides with the true average bounding box, which is the specific range of the average bounding box manually framed during labeling.

For the structured road features of highways, this paper completes the original point cloud ground segmentation process based on two segmentation methods, namely, ray slope threshold and random sampling consistency-based planar model. Comparing the results of the two methods, many ground point clouds can be filtered out, and the morphological information of the road boundary and the vehicles within the road is retained completely. The segmentation method based on ray slope threshold can adjust the segmentation threshold according to the point cloud position, which can effectively avoid oversegmentation and undersegmentation, and apply this method to the environment perception system of ADAS. The KD-tree search method is used to cluster the detected targets based on Euclidean distance, multiple clustering threshold regions are divided for the LIDAR point cloud density characteristics, and the target vehicle location and size information is stored in the 3D rectangle after clustering processing. The tracking test results show that the algorithm can continuously track the target and meet the requirements of behavioral decision and motion planning control system for sensory information.

RETRACTED

### 4.2. System Performance Analysis

The ACC function designed in this paper is applied to the cruise control of L3 autonomous vehicles, and the ACC function is tested according to ISO/NP 22179 test protocol published by the International Organization for Standardization. The core function of ACC is to allow the autonomous vehicle to maintain a safe distance from the target vehicle in front and to follow the vehicle in front for cruise control. To verify the functional requirements of ACC, the corresponding test conditions are designed as shown in Figure 7, with the reference vehicle speed being the same as the initial speed.

The initial distance is within the safe distance. When the initial speed of the self-driving vehicle is greater than the target vehicle, the self-driving vehicle starts to decelerate within 0 ∼ 2 S. When the speed of the self-driving vehicle decreases below the speed of the target vehicle and the distance between the two vehicles does not reach the safe distance, the ACC system maintains the deceleration following state, and the simulation time lasts for 6 S. When the distance between the two vehicles exceeds the safe distance, the self-driving vehicle enters the acceleration following state. In 6∼12 s time, the speed of the two vehicles gradually reaches equal to the speed of the two vehicles gradually. Since the target vehicle is driving with a small acceleration of 0.1 m/s^2^, which leads to a small overshoot of the autonomous vehicle speed tracking, the speed tracking effect is optimized by adjusting the PID controller parameters or increasing the dead zone in a small range.

From Figure 8, we get the position information of the autonomous vehicle and the right adjacent lane vehicle in the global reference coordinate system; there is no *y*-direction movement of the vehicle during the simulation, so the vertical coordinate in the figure is the position of the vehicle in the *x*-direction. The initial position of the autonomous vehicle (0, 0) is along the positive direction of the *x*-axis, and the position of the right vehicle is (32, −3.5); both vehicles are driving in the same direction, and the lane width is 3.5 m. At 385 m, from the origin, the autonomous vehicle overtakes the right vehicle and completes the tracking test. According to the test results, the ACC system can accurately detect the target vehicle, control the autonomous vehicle to follow the speed of the target vehicle well, complete the acceleration and deceleration actions, and maintain a safe driving distance.

RETRACTED

The simulation results show that the autonomous vehicle decelerates slowly first. When the simulation time is 4s, the target vehicle 1 starts to change lanes, and the speed of the target vehicle jumps to zero, and there is a small fluctuation. When the stationary target vehicle 2 in front is detected, the distance and safety distance between the two vehicles suddenly change. With the acceleration of the target vehicle 2, the distance between the two vehicles changes slowly. Before reaching the safety distance, the autonomous vehicle speed decreases to the speed value of the target car 2 and continues to maintain the safety distance to follow the car. From the test results, it is concluded that the ACC function can realize the repositioning of the tracking target, which can meet the demand of switching the tracking target during the cruising process. There is a delay of 1 s in the system control of vehicle speed after switching targets in the figure, but the perception information is accurate, and the reason is analyzed to be the real-time problem of data transfer between perception information and decision system, which will be improved in the subsequent research work.

As can be seen, the binocular visual ranging algorithm requires stereomatching to calculate the parallax in the two parallax maps, which increases the amount of computation and seriously reduces the speed of range, and can only process five frames per second when using the SGBM algorithm for stereomatching. Therefore, this chapter adopts the monocular vision ranging method, which relies entirely on mathematical models, with fast computation speed and small model size. However, the difference between the detection accuracy and binocular vision is still relatively large, especially for long-distance targets. At the same time, the monocular vision ranging method also requires presetting most of the values in the mathematical model and calibrating the vision sensor, which requires some preparation work before use. There is almost no requirement for distance measurement for long-range targets, and the monocular vision ranging approach is more in line with the needs of this paper's topic with faster detection speed and a relatively simple mathematical model that only needs to extract one feature point for distance detection. After getting the distance information, the decision-making mechanism of the assisted driving system can determine and make decisions on the dangerous information present in the surrounding environment; i.e., the assisted driving algorithm can sense danger.

RETRACTED

## 5. Conclusion

1. This paper uses a lightweight neural network to reduce the complexity of the faster R-CNN algorithm and then links it with a relatively simple monocular vision ranging model, which can be used in the range of 50 meters. It depends on the flexibility and generality brought by the pure mathematical model. It can be said that monocular vision ranging method is the first choice of assisted driving algorithm.
2. This paper proposes a target depth estimation algorithm based on classification, that is, width estimation algorithm. The algorithm obtains a structured understanding of the vehicle target through the cluster analysis of the appearance of the vehicle rearview mirror. The algorithm improves the traditional image processing method, so it can be applied to multitask neural network.
3. Theoretical calculation and field experiments verify the effectiveness and stability of the algorithm. The traditional image segmentation method and depth estimation network segmentation method are compared and analyzed, and the results show that the algorithm is more accurate. The depth estimation algorithm of the learning model and other tasks can be integrated into multiple target regions at the same time.
4. In the MPC based path planner, the vehicle model is linearized and used to solve the objective function to realize the dynamic path replanning function. A path tracking controller based on MPC algorithm is designed to dynamically control the front wheel angle through the rolling optimization strategy, so that the tracking error of the autonomous vehicle on the expected path meets the constraints, and the speed control selects the response PID controller, effectively controlling the throttle opening and the braking pressure required to reach the required speed.

## Figures and Tables

**Figure 1:** Principal diagram of improved R-CNN.

**Figure 2:** Transformed image after Hough transform.

**Figure 3:** Software design scheme.

**Figure 4:** Accuracy of different detection algorithms.

**Figure 5:** Model length and width distribution.

**Figure 6:** Comparison of backbone networks.

**Figure 7:** ACC test conditions.

**Figure 8:** Simulation results of following the target vehicle.

## Data Availability

The figures used to support the findings of this study are included in the article.
